# Amino acid synthesis loss in parasitoid wasps and other hymenopterans

**DOI:** 10.7554/eLife.59795

**Published:** 2020-10-19

**Authors:** Xinhai Ye, Shijiao Xiong, Ziwen Teng, Yi Yang, Jiale Wang, Kaili Yu, Huizi Wu, Yang Mei, Zhichao Yan, Sammy Cheng, Chuanlin Yin, Fang Wang, Hongwei Yao, Qi Fang, Qisheng Song, John H Werren, Gongyin Ye, Fei Li

**Affiliations:** 1 State Key Laboratory of Rice Biology & Ministry of Agricultural and Rural Affairs Key Laboratory of Molecular Biology of Crop Pathogens and Insects, Institute of Insect Sciences, Zhejiang UniversityHangzhouChina; 2 Department of Biology, University of RochesterRochesterUnited States; 3 Division of Plant Sciences, College of Agriculture, Food and Natural Resources, University of MissouriColumbiaUnited States; Vanderbilt UniversityUnited States; University of MichiganUnited States

**Keywords:** amino acid synthesis, trait loss, comparative genomics, genome sequencing, parasitoid wasps, Cotesia chilonis, Other

## Abstract

Insects utilize diverse food resources which can affect the evolution of their genomic repertoire, including leading to gene losses in different nutrient pathways. Here, we investigate gene loss in amino acid synthesis pathways, with special attention to hymenopterans and parasitoid wasps. Using comparative genomics, we find that synthesis capability for tryptophan, phenylalanine, tyrosine, and histidine was lost in holometabolous insects prior to hymenopteran divergence, while valine, leucine, and isoleucine were lost in the common ancestor of Hymenoptera. Subsequently, multiple loss events of lysine synthesis occurred independently in the Parasitoida and Aculeata. Experiments in the parasitoid *Cotesia chilonis* confirm that it has lost the ability to synthesize eight amino acids. Our findings provide insights into amino acid synthesis evolution, and specifically can be used to inform the design of parasitoid artificial diets for pest control.

## Introduction

The Hymenoptera contain diverse insects (e.g. sawflies, wasps, bees, and ants) which utilize a wide variety of food resources (Quicke, 1997; Peters et al., 2017). Among the Hymenoptera, parasitoids account for about 75% of species and 10 ~ 20% of all insect species (Pennacchio and Strand, 2006). They are also important biological control agents in integrated pest management (IPM) (Bale et al., 2008). Female parasitoid wasps attack arthropod hosts and lay their eggs upon (ectoparasitoid) or within (endoparasitoid) them, where the offspring feed and develop, eventually causing host death. Therefore, parasitoids feed on a food resource rich in proteins, lipids, and other nutrients. In addition, parasitoids can manipulate the nutritional value of the hosts through effectors injected into the host, such as venom proteins, polydnaviruses, and molecular factors produced by parasitoid cells (teratocytes) that are either injected into the host or produced by feeding larvae (Pennacchio and Strand, 2006; Pennacchio et al., 2014). As well as inhibiting host immunity and alterning host development, these mechanisms alter host metabolism in ways that mobilize nutrients from host tissues to meet the demands of developing larvae (Mrinalini et al., 2015; Pennacchio et al., 1995; Rivers and Denlinger, 1994).

We originally began this project to investigate how the protein-rich diet of parasitoids and their ability to manipulate amino acid availability in hosts, has affected their genomic repertoire in amino acid synthesis pathways. Our hypothesis was that parasitoids would show extensive loss of genes in amino acid synthesis pathways due to the availability of amino acids in their diet.

Gene loss in nutritional biosynthetic pathways has been described in several insect groups. For instance, some hemipteran insects have lost genes in amino acid biosynthetic pathways, apparently because they can obtain the nutrition from their endosymbionts (Douglas, 2006; Feldhaar, 2011). In some cases, this has been confirmed by annotation of the complete pathway of the endosymbiont and incomplete pathway of the insect, for instance in aphids (Richards et al., 2010), planthoppers (Xue et al., 2014), leafhoppers (McCutcheon and Moran, 2007), and mealybugs (Husnik and McCutcheon, 2016; Gil et al., 2018). Many of these studies involve herbivorous insects that feed on plant sap. However, hymenopteran insects have diverse food resources. Thus, it is reasonable to assume that changes involved in some biosynthetic pathways occurred during the evolution of hymenopteran insects. In particular, carnivorous parasitoid wasps feed on a protein and lipid-rich food resource of hosts, which could have resulted in genomic changes. This prompted us to investigate whether some gene losses occur in the nutritional biosynthetic pathways and how parasitoid wasps exploit the nutrition of hosts.

The amino acid, carbohydrate, and lipid requirements of several parasitoid wasps have been evaluated using the traditional nutrient removal method (Thompson, 1986), that is removing particular components from an artificial diet. Parasitoid wasps can manipulate their hosts to produce a nutritionally favorable environment for parasitoid development, and there is considerable evidence that they do so through venoms and teratocytes injected by the mother into the host and via modifications induced by feeding larvae (Nakamatsu and Tanaka, 2003; Nakamatsu and Tanaka, 2004; Pennacchio et al., 2014). For example, parasitoid venoms induce a higher concentration of lipids, which is confirmed by in vitro injection of venom into the host (Nakamatsu and Tanaka, 2003; Nakamatsu and Tanaka, 2004). Detailed transcriptomic and metabolomic analyses of venom injected hosts of *Nasonia vitripennis* reveal dramatic alterations in host gene expression (Martinson et al., 2014), sugar, chitin, and lipid metabolism, as well as elevation of free amino acid levels (Mrinalini et al., 2015). To meet the demands of the developing wasp larvae, nutritional components such as proteins, acylglycerols and free amino acids change in the hemolymph of the parasitized pea aphid *Acyrthosiphon pisum* during development of parasitoid wasp *Aphidius ervi* larvae (Pennacchio et al., 1995; Rahbé et al., 2002). Previous studies showed that at early stages, endoparasitoid wasp larvae absorb nutrients from host hemolymph through thin exoskeletons and epidermis, whereas they absorb nutrients mainly through gut epithelium at later stages (Giordana et al., 2003; Caccia et al., 2005; Grimaldi et al., 2006; Pennacchio et al., 2014). Although parasitoids develop on a nutritionally rich food resource and manipulate the nutritional qualities of the host, there have been very few studies on how this relationship impacts their genomic evolution. Although some studies have investigated lipid utilization and biosynthesis in parasitoids (Visser and Ellers, 2008; Visser et al., 2010; Visser et al., 2012; Lammers et al., 2019), there has been very little research on changes in amino acid biosynthetic pathways.

To investigate the idea that parasitoids have lost essential amino acid synthesis genes due to their amino-acid-rich food resource, we first conducted genome sequencing of *Cotesia chilonis* and examined its genomic repertoire for amino acid synthesis pathway genes. To place these results in an evolutionary context, we next examined the genomes of 38 hymenopteran species (3 sawflies, 17 aculeates and 18 parasitoids) for which well assembled and annotated genomes are available, and compared these to a set of 13 other holometabolous and hemimetabolous arthropods. We then returned to *C. chilonis* to conduct a set of experiments to investigate the amino acid requirements of their larvae, in light of the pathways predicted to be disrupted by the genomic analysis. To investigate the effects of parasitoid venom and feeding larvae on host amino acids, changes in these host nutrition components in host hemolymph were analyzed after parasitism by this wasp, using UPLC-MS/MS (ultra‐performance liquid chromatography tandem mass spectrometry). Finally, the in vitro deletion method was used to determine which essential amino acids developing wasps require from its host.

Here, we consider three kinds of losses relevant to amino acid metabolism: gene loss in amino acid pathways, pathway disruption due to gene loss, and loss of synthesis ability for different amino acids. It is noteworthy that pathway disruption for a particular amino acid does not always mean loss of the ability to synthesize that amino acid, because there are alternative pathways for synthesis of some amino acids. Our results indicate a disruption of 16 amino acid pathways at the base of the branch leading to holometabolous insects, which disrupted the synthetic capability for four amino acids (tryptophan, phenylalanine, tyrosine and histidine). Additional disruption of seven pathways occurred basally in the Hymenoptera, which caused the loss of synthesis capability for three additional amino acids (valine, leucine, and isoleucine). The result indicates that hymenopterans have lost the ability to synthesize seven amino acids. Subsequently during the evolution of Hymenoptera, independent pathway disruptions related to the biosynthesis of two amino acids (lysine and cysteine) were found. The lysine pathway disruptions caused several independent losses of synthesis capability for lysine both in members of the Aculeate and Parasitoida infraorders. The disruptions in the cysteine pathway were only found in the Parasitoida infraorder, and they did not disrupt the synthesis capability of cysteine because alternative pathways for cysteine synthesis remained. *C. chilonis* shows the seven expected amino acid synthesis losses in Hymenoptera, based on the phylogenetic analysis, and an additional loss of lysine synthesis found in *C. chilonis* and close relatives relative to other hymenopterans. Our nutritional experiments show that *C. chilonis*, as expected, has lost the ability to synthesize these eight amino acids.

## Results

### Genome evolution of *C. chilonis*

The evolution of hymenopteran insects has attracted increasing research interest. Many phylogenetic analyses have been conducted using transcriptome data (Bank et al., 2017; Peters et al., 2017; Peters et al., 2018). Since genomic sequences contain more information than transcriptomes, we used the available hymenopteran genomes to infer the phylogenetic relationships between *C. chilonis* and 13 other hymenopteran species (8 parasitoids and 5 non-parasitoids). The protein sequences of 2291 single-copy genes were used for phylogenetic inference and the red flour beetle *Tribolium castaneum* was used as the outgroup. Phylogenetic analysis by the maximum likelihood phylogenetic method showed that *C. chilonis* clusters with four braconid wasps, as expected, to form a group in the family Braconidae, a member of the superfamily Ichneumonoidea (Figure 1B). As previously established (Heraty, 2009; Misof et al., 2014; Peters et al., 2017), the superfamily Ichneumonoidea is a sister group to the superfamily Chalcidoidea, and the parasitoid wasps in Braconidae and Chalcidoidea are clustered together, and are members of the infraorder Parasitoida (Peters et al., 2017), which is a sister group to the infraorder Aculeata (containing vespid wasps, ants, and bees). The Parasitoida contains a number of superfamilies in addition to the Ichneumonoids and Chalcidoids, such as Cynipoids, Platygastroids, and Protrotrupoids. Most species are parasitoids, with some reversions to plant feeding, such as in some cynipoids and in pollinating fig wasps (Heraty, 2009; Peters et al., 2017).

**Figure 1.** Hymenoptera genome evolution and comparative genomic analysis. (**A**) A female *C. chilonis* attacking its host *C. suppressalis* and the cocoons of *C. chilonis*. (**B**) Hymenoptera phylogeny and orthology assignment based on genome data. The phylogenetic tree was based on 2291 single-copy proteins. Red flour beetle *T. castaneum* was used as the outgroup. Divergence time for each node is represented by gray bars at the node, the range of the bar indicated the 95% confidence interval of the divergence time. Bars are subdivided to represent different types of orthology clusters, as indicated. Universal single-copy genes are single-copy across all species analyzed by us, and absence or duplication in a single genome was allowed; Universal multiple-copy genes represent other universal genes; Specific duplication represents specific duplication genes; Species-specific genes represent species-specific genes with only one copy in the genome; Dispensable clusters represent the remaining genes. (**C**) Amino acid identity of pairwise species. (**D**) Gene collinearity analysis between three braconid wasps (using scaffolds that contain more than five genes) with MCScanX. The heavy bars represent all the scaffolds linked together in an artificial order. In *C. chilonis* and *M. demolitor* pair, 6335 genes constituted 497 synteny blocks; In *C. chilonis* and *M. cingulum* pair, 946 genes constituted 127 synteny blocks. Figure 1—source data 1.This file includes the phylogeny tree file in Figure 1B. Figure 1—source data 2.This table includes the orthology assignment based on genome data. Figure 1—source data 3.This table includes the amino acid identity of pairwise species. Figure 1—source data 4.This table includes the gene collinearity pairs among *C. chilonis*, *M. cingulum* and *M. demolitor*.

*C. chilonis *has a close relationship with another braconid wasp, *M. demolitor*, with 75% amino acid identity in orthologous proteins (Figure 1C). We chose scaffolds that contain more than five genes for synteny analysis among three braconid wasps, and found that chromosomal rearrangement frequently occurred in various wasp species, especially after the divergence of *C. chilonis* and *M. cingulum* (Figure 1D). *C. chilonis* was estimated to have diverged from *M. demolitor* approximately 61.05 (31.74–108.70) million years ago.

### Disruptions in amino acid biosynthetic pathways in hymenoptera

We next conducted a comparative analysis in hymenopterans for gene loss and pathway disruptions in amino acid biosynthesis (Figure 2, Figure 3), and loss of synthesis capability for different amino acids (Figure 2C). KEGG modules (or sub-pathways) for amino acid biosynthesis were used for our analyses, which were also used in the pathway study of parasitic worms (Coghlan et al., 2018). We define a pathway disruption as the loss of one or more genes required for amino acid synthesis in the pathway. The loss of synthesis capability to an amino acid occurs when all synthetic pathways for this amino acid are disrupted in such a way that there is no complete path to synthesis of the amino acid based on the currently known pathways. It should be noted that the pathway disruption and loss of synthesis capability are different, because there are alternative pathways for synthesis of some amino acids.

**Figure 2.** Pathway disruptions and independent gene losses in the amino acid biosynthetic pathways and loss of amino acid biosynthetic capability in Hymenoptera. (**A**) Phylogenetic tree of 38 hymenopteran insects and pathway disruptions during the Hymenoptera evolution. In total, we have documented 14 independent disruptions of the amino acid synthetic pathways in hymenopterans, 10 in Ichneumonoid/Chalcidoid clade and four in the Aculeata clade. These independent pathway disruptions were showed as triangles on the branches. (**B**) Independent gene losses in amino acid biosynthetic pathways (white, present; black, lost). In Hymenoptera, 164 independent gene losses were found, 77 in the Chalcidoid/Ichneumonoid clade and 63 in the Aculeate clade. (**C**) Amino acid biosynthetic capability of each species was evaluated in terms of combined metabolic pathways for each amino acid (white, present; black, lost). The most recent common ancestor (MRCA) states of Hymenoptera (HYM) and Holometabola (HOL) were reconstructed using 13 additional outgroups to Hymenoptera. Figure 2—source data 1.This file includes the phylogeny tree file in Figure 2A. Figure 2—source data 2.Genes in amino acid biosynthetic pathways, '+' means present, 'x' means lost. Figure 2—source data 3.Amino acid biosynthetic capability of each species, '+' means present, 'x' means lost.

**Figure 3.** Amino acid biosynthetic pathways that have been disrupted in the most recent common ancestor (MRCA) of Holometabola, MRCA of Hymenoptera, MRCA of Braconidae and MRCA of *Cotesia*. We defined a pathway disruption as the loss of one or more genes required for amino acid synthesis in the pathway (KEGG modules). The KEGG modules in black box mean the novel disruptions compared to the outgroups. The amino acid biosynthetic pathways are redrawn from KEGG pathway, map01230. The gene losses caused the pathway disruptions during the Hymenoptera evolution are shown in colorful arrows, corresponding to the pathway disruption events shown in Figure 2A.

Two major superfamilies of parasitoid wasps, Ichneumonoidea and Chalcidoidea (in the infraorder Parasitoida, Peters et al., 2017) were examined, along with members of the infraorder Aculeata. Species were selected that have well-assembled genomes. For Parasitoida, there are 2 in the Ichneumonidae, 8 in the Braconidae, and 7 in the Chalcidoidea. For the Aculeata, there is 1 paper wasp (Vespidae), 8 ants (Formicidae), and 8 bees (Anthophila). Both of these infraorders have additional superfamilies, but we focused our analysis on this set because they have high-quality genome assemblies, which are necessary for reliable identification of gene loss. The more basal hymenopteran sawflies *A. rosae* (Tenthredinoidea), *Neodiprion lecontei* (Tenthredinoidea), *Cephus cinctus* (Cephoidea), and parasitic wood wasp *O. abietinus* (Orussoidea) were also used for comparisons. In total, 10 ichneumonoid wasps, 7 chalcidoid wasps, 1 paper wasp, 8 ants, 8 bees, 1 parasitic wood wasp, and 3 sawflies were included in this analysis. In addition, to learn more about the ancestral state of Hymenoptera, we used 13 species in orders outside of Hymenoptera (2 from Coleoptera, 2 from Lepidoptera, 3 from Diptera, 2 from Hemiptera, 1 from Thysanoptera, 1 from Collembola, and 1 each from arthropod taxa Cladocera and Trombidiformes) to evaluate the ancestral amino acid synthesis repertoire (Supplementary file 1 – Table 1).

After filtering potential contaminated bacterial sequences using a pipeline modified from Wheeler et al., 2013 (see Materials and methods), the BlastKOALA web server and iPathCons tool were used to reconstruct the amino acid biosynthetic pathway in each genome. For each species, we identified losses of genes and pathway disruptions in the pathways and synthesis capability to amino acids (Figure 2, Supplementary file 1 – Table 1). The ancestral amino acid biosynthetic pathways of Hymenoptera, holometabolous insects were constructed based on the gene losses in the pathways and species phylogenetic positions.

Pathway disruption is not the same as a loss of capability to synthesize an amino acid, because alternative pathways are available for some amino acids (Figure 2). We first examined gene losses, pathway disruptions, and amino acid synthesis loss in the species set (Figure 2A, Figure 2B, Supplementary file 1 – Table 1). Seven pathway disruptions and 16 gene losses have occurred in the common ancestor of Hymenoptera (Figure 2B, Figure 3) after their divergence from other holometabolous insects. These disrupted pathways are related to synthesis of cysteine (M00021 and M00609), valine/leucine/isoleucine (M00019, M00432 and M00570) and arginine (M00844 and M00029).

Within the Hymenoptera, we have documented 14 independent disruptions of the amino acid synthetic pathways, 10 in the Ichneumonoid/Chalcidoid clade and 4 in the Aculeata clade, based on the genes involved and phylogenetic position of the species (Figure 2A). Both aculeates and parasitoids show pathway disruptions in amino acid biosynthesis. There is no significantly difference between the observed proportion of pathway disruptions in the Ichneumonoid/Chalcidoid clade (71%) and the expected proportion (55%) (p=0.695, Fisher’s exact test, N = 14).

We also compared the frequency of gene losses within pathways, and identified a total of 164 independent gene losses, 63 in the Aculeate clade and 77 in the Chalcidoid/Ichneumonoid clade (Figure 2B, Supplementary file 1 – Table 1). The number of independent gene losses is higher than the number of independent pathway disruptions in Hymenoptera evolution. This is mainly due to two reasons: (1) there are many gene losses in the pathways which had already been disrupted in the common ancestor of Hymenoptera or earlier; (2) there can be more than one gene loss in the same pathway during the Hymenoptera evolution. Total gene losses show a similar frequency between the Ichnuemonoid/Chalcidoid and Aculeate clades based on branch lengths (55% observed vs 55% expected compared to 45% vs 45% expected (p=1, Chi-square test, Supplementary file 2 – Table 1)), indicating that neither clade is enriched for gene losses relative to the other.

Three pathways (M00030, M00433 from lysine synthetic pathways and the pathway from 3-phosphoserine to cysteine) were disrupted during hymenopteran evolution in some lineages, with 14 independent events (Figure 2A, Figure 3). Loss of M00030 is the direct cause of loss of capability to synthesize lysine, which independently happened nine times in Hymenoptera, five in the Ichneumonoid/Chalcidoid clade and four in the Aculeata clade. All these are due to loss of the same gene in the M00030 pathway, aromatic amino acid aminotransferase I [EC:2.6.1.57 2.6.1.39 2.6.1.27 2.6.1.5] (ARO8, K00838) (Figure 2B, Figure 3). In the Ichneumonoidea, the *ARO8* gene was lost in nine wasps, but retained in the braconid wasp *Fopius arisanus*. Their phylogeny positions suggest there are four independent loss events (Figure 2A). This gene can be found in the earlier branch of Chalcidoidea, *Trichogramma pretiosum*, but cannot be detected in any other chalcidoid wasps in this analysis. This result suggests a gene loss event in the common ancestor of six chalcidoid wasps (Figure 2A). In the eight ants in this analysis, this gene was lost in four ants, including *Harpegnathos saltator*, *Solenopsis invicta*, *Atta cephalotes* and *Acromyrmex echinatior*. This result suggests that this gene was independently lost in the *H. saltator* and the common ancestor of *S. invicta*, *A. cephalotes* and *A. echinatior* (Figure 2A). In bees, two independent losses of this gene were found in the *Dufourea novaeangliae* and the common ancestor of *Eufriesea mexicana*, *Apis mellifera*, *Melipona quadrifasciata* and two *Bombus* bees (Figure 2A). The pattern suggests that this gene is prone to independent loss during evolution. Another lysine biosynthetic pathway module (M00433) was independently lost in the ichneumonid wasp *Venturia canescens* and braconid wasp *Aphidius ervi* due to the loss of homocitrate synthase [EC:2.3.3.14] (LYS21, K01655). This gene can be found in many other hymenopteran insects in this analysis (Figure 2A). Disruption of M00433 only happened in parasitoid wasps, and occurred after lysine synthesis capability was lost due to disruption of the M00030 pathway. We also identified another gene, cysteine synthase [EC:2.5.1.47 2.5.1.65 4.2.1.22] (cysO, K10150) that converts 3-phosphoserine to cysteine, which was independently lost in the *V. canescens*, the common ancestor of two aphid parasitoids (*A. ervi* and *Lysiphlebus fabarum*) and the common ancestor of four pteromalid wasps (Figure 2). However, loss of *cysO* doesn’t disrupt the cysteine biosynthesis because cysteine can be converted from L-cystathionine by cystathionine gamma-lyase [EC:4.4.1.1] (CTH, K01758) in M00338 (Figure 3).

During the evolution of Hymenoptera, we found many gene losses in pathways which had already been disrupted in the common ancestor of Holometabola and the common ancestor of Hymenoptera. Examples include the synthetic pathway for histidine (M00026) and aromatic amino acids (M00024 and M00025). Examination of pathway completeness for seven species from three different orders of Holometabola (Coleoptera, Lepidoptera, and Diptera) revealed that 16 pathways were disrupted in the common ancestor of Holometabola (causing loss of biosynthesis in four amino acids). Seven pathways were newly disrupted in the Hymenoptera after their divergence from other holometabolous insects (Figure 3), leading to a synthesis loss for three amino acids. There is a total of 125 (76%) independent gene losses in Hymenoptera for pathways that had already been disrupted in the common ancestor of Holometabola. This is significantly higher than the random expected proportion of gene losses (52%) estimated based on the gene number of each pathway in the ancestral state of Hymenoptera (p<0.01, *df* = 2, Chi-square test, Supplementary file 2 – Table 2). This pattern is expected, given that once the pathway is disrupted, selection to maintain other genes in the pathway would be diminished, unless the gene had functions in other pathways as well. Indeed, the persistence of some genes in these pathways implies that they have other functions that have resulted in their retention in evolution. Only 15 (9%) of independent gene losses occurred in pathways that had been disrupted in the common ancestor of Hymenoptera, which is lower than the expected proportion of 30%. Twenty-four (15%) independent gene losses happened in the pathways that were functional in the common ancestor of Hymenoptera, which is similar to the expected proportion of 18%. This result suggested that gene losses are more likely to occur in pathways which have already been disrupted in the common ancestor of Holometabola.

We also compared the gene losses between the Ichnuemonoid/Chalcidoid and Aculeate clades, in the pathways that are complete in the common ancestor of Hymenoptera. We documented 17 independent gene loss events in the Ichnuemonoid/Chalcidoid clade and 6 in the Aculeate clade. There is no significant difference between the observed proportion of pathway disruptions in the Ichneumonoid/Chalcidoids (74%) and the expected proportion (55%) based on branch lengths (see Materials and methods) (p=0.207, Chi-square test, Supplementary file 2 – Table 3). As more well-assembled genomes come available for these taxa, the question can be revisited.

### Changes in amino acid synthesis capability in the hymenoptera

A disruption of an individual pathway does not necessarily lead to loss of amino acid synthesis capability, due to redundancy in pathways for some amino acids. Based on the pathway completeness (i.e. coverage of reference pathway in KEGG, map01230), we next evaluated how the capability to synthesize amino acids has changed during evolution. Hymenoptera is the basal order for the holometabolous insects (Savard et al., 2006; Misof et al., 2014). The capabilities to synthesize histidine, tryptophan, tyrosine, and phenylalanine appear to have been lost early in holometabolous insects, prior to divergence of the basal Hymenoptera (Figure 2C). The capabilities to synthesize valine, leucine, and isoleucine were subsequently lost in the common ancestor of Hymenoptera after their divergence from other holometabolous insects (Figure 2C). This was due to the losses of two key genes in the valine/leucine/isoleucine pathway, ketol-acid reductoisomerase [EC:1.1.1.86] (ilvC, K00053) and acetolactate synthase I/III small subunit [EC:2.2.1.6] (ilvH, K01653) (Figure 2B). As a result, our data show that synthesis capability of four amino acids (tryptophan, phenylalanine, tyrosine, and histidine) was lost earlier in holometabolous insects, and synthesis capability of three amino acids (valine, isoleucine and leucine) was lost in the common ancestor of Hymenoptera. Otherwise, the capability to synthesize amino acids in Hymenoptera is largely conserved, despite the disruptions of three pathways with 14 independent events. This is due to the redundancy in synthesis for certain amino acids. We only detected losses of the capability to synthesize lysine within different lineages of hymenopterans, all of which are due to independent gene loss in the same gene, *ARO8* (K00838) in the M00030 pathway. After the loss of capability to synthesize lysine caused by disruption of M00030, a gene in the M00433, *LYS21* (K01655), was lost independently in ichneumonid wasp *V. canescens* and braconid wasp *A. ervi* (Figure 2A). In this analysis, 25 hymenopteran species lost the capability to synthesize lysine, 15 in the Ichneumonoid/Chalcidoid clade and 10 in the Aculeata clade (Figure 2C). Their phylogeny positions suggest these are due to nine independent loss events, five in the Ichneumonoid/Chalcidoid clade and four in the Aculeata clade. We did not find synthesis loss in *Orussus* or the sawflies. Disruptions of the pathway from 3-phosphoserine to cysteine in some parasitoid lineages caused by single gene loss does not disrupt the cysteine biosynthesis because it can be converted from L-cystathionine by *CTH* (K01758) in M00338 (Figures 2 and 3). These are in addition to the disruption of 7 amino acid pathways (which resulted in synthesis capability loss of valine, leucine and isoleucine) in the common ancestor of the Hymenoptera, and 16 pathway disruptions in the common ancestor of the Holometabola (which resulted in synthesis capability loss of histidine, tryptophan, tyrosine, and phenylalanine). Therefore, different hymenopteran species in our data set show a total of 23–26 pathway disruptions, depending on whether loss of the lysine (M00030, M00433) or/and cysteine (from 3-phosphoserine to cysteine) pathways occurred within its lineage. The number of synthesis capability losses ranged from seven to eight, depending on whether lysine synthesis capability, due to disruption in the lysine pathway M00030, occurred in a particular lineage.

In *C. chilonis*, our analysis showed 24 pathway disruptions, 23 of them occurred basally in Hymenoptera or earlier, and the remaining one (M00030) happened in the common ancestor of *Cotesia*, *Microplitis* and *Macrocentrus.* These pathway losses disrupted the biosynthesis of eight amino acids (lysine, tryptophan, phenylalanine, tyrosine, isoleucine, leucine, valine, and histidine) (Figure 4A, Supplementary file 2 – Table 4, Table 5). We next examined this result by amino acid depletion feeding assays and confirmed for all eight in this study (see below).

**Figure 4.** *C. chilonis* loses the ability to synthesize eight amino acids. (**A**) Gene loss in amino acid biosynthetic pathways in *C. chilonis*. BlastKOALA web server and iPathCons tool were used for re-constructing the amino acid biosynthetic pathway in *C. chilonis* with annotated *C. chilonis* protein coding genes. For those genes missing in the first step, we searched them in whole genome assembly and PacBio long reads by TBLASTN (see Materials and methods). In total, 46 genes were found to be missing in the amino acid biosynthesis pathway for *C. chilonis*, thus disrupting the biosynthesis of eight amino acids (Lys, Trp, Phe, Tyr, Ile, Leu, Val, His). Full line indicates the reaction exists in *C. chilonis*, while dotted line indicates the interaction cannot be found. Amino acid names in red can be synthesized by *C. chilonis*, names in gray with strikethrough cannot be synthesized due to the lost genes on each dotted line. (**B**) In vitro rearing of *C. chilonis*. Five days after parasitism, larvae were put on the membrane of a transwell chamber; then the transwell was placed in the well containing 250 μl of *Cotesia* rearing medium so that the wasp larvae could reach the nutrients (see Materials and methods). (**C**) Survival rates of *C. chilonis* larvae developed on 11 different rearing media, respectively. Positive control: Grace's Insect Medium, containing 20 amino acids (see Materials and methods, *n* = 30); Negative control uses positive control medium minus the eight amino acids that *C. chilonis* cannot synthesize, Lys, Trp, Phe, Tyr, Ile, Leu, Val, His, *n* = 30; Single amino acid deficiencies use control media minus only one amino acid, indicated by '-' superscript, for example Gly deficiency (Gly^-^) indicates excluding glycine only. Gehan-Breslow-Wilcoxon test was used for survival rate statistical analyses. The Benjamini-Hochberg method was used for multiple testing correction. The statistical results of pairwise group comparisons are indicated. Figure 4—source data 1.Genes in amino acid biosynthetic pathways of *C. chilonis*. Figure 4—source data 2.This table includes the survival rates of *C. chilonis* larvae developed on 11 different rearing media.

**Figure 4—figure supplement 1.** Activation of amino acid biosynthetic pathways. Threonine (**A**), arginine (**B**), and methionine (**C**) are generally regarded as essential amino acids in *C. chilonis*, while alanine (**D**) and serine (**E**) are non-essential amino acids. The gray arrows mean the gene loss. Gene expression at different development stages (from left to right, early larvae, later larvae, female pupa, male pupa, female adult, and male adult) as measured by quantification of transcription levels (log2FPKM) is shown in the histograms.

### Loss of the ability to synthesize eight amino acids in *C. chilonis*

Although many efforts have been devoted to elucidate the immune manipulation of hosts by parasitoid wasps, relatively less is known about the nutrition interactions between the host and parasitoid (Pennacchio et al., 2014). A high-quality genome of the host *C. suppressalis* has previously been reported (Yin et al., 2014; Ma et al., 2020), so *C. chilonis-C. suppressalis* is an excellent model system to investigate the genetic basis of nutrition utilization of the host by parasitoid wasps, and its implications to gene gains and losses in the parasitoid. Our analysis above has shown that the *C. chilonis* has experienced pathway and gene losses in its evolutionary history that have disrupted the biosynthesis of eight amino acids (lysine, tryptophan, phenylalanine, tyrosine, isoleucine, leucine, valine, and histidine) (Figure 4A, Supplementary file 2 – Table 4, Table 5). All these are essential amino acids for parasitoids except tyrosine, which can be synthesized from phenylalanine (Thompson, 1981). The genes related to the biosynthesis of three other essential amino acids (arginine, methionine and threonine) were not lost. For methionine and threonine, although the biosynthetic pathways from aspartate were broken by some gene loss, these amino acids can be synthesized from another non-essential amino acid, serine (Figure 4—figure supplement 1). The expression of genes in the pathway from serine to methionine and threonine also were examined using RNA-seq data, and it was found that all genes could be expressed in at least one stage during wasp development. Interestingly, the 5-methyltetrahydrofolate-homocysteine methyltransferase (metH; EC: 2.1.1.13) gene in the last step to synthesize methionine was only expressed in later larvae and adults, which means *C. chilonis* cannot synthesize methionine by itself in early larval and pupal stages (Figure 4—figure supplement 1). For arginine, the biosynthetic pathway from glutamate to arginine (KEGG module: M00845) was broken, but the pathway from ornithine to arginine (KEGG module: M00844) was complete with gene expression at different life stages (Figure 4—figure supplement 1). These results indicate that, from a genomic point of view, *C. chilonis* can synthesize arginine, threonine, and methionine (but for methionine, only at later larval and adult stages).

### In vitro verification of requirements for different amino acids

To study how the loss of the capability to synthesize certain amino acids influences larval development, we in vitro reared 5-day-old *C. chilonis* larvae in the chemically defined medium (Figure 4B; see Materials and methods). The Grace's Insect Medium (see Materials and methods for detail components and concentrations), which contains 20 amino acids was used as a positive control, and the baseline medium which deleted eight amino acids (lysine, tryptophan, phenylalanine, tyrosine, leucine, isoleucine, valine, and histidine) that *C. chilonis* cannot synthesize based on the genomic analysis, was used as a negative control. In addition, eight different media with exclusion of each individual amino acid were also tested. The results indicated that the absence of any of the eight amino acids mentioned above led to developmental arrest of parasitoid larvae, demonstrating that *C. chilonis* larvae cannot survive in the medium without each of these eight amino acids. However, they could survive in the medium without glycine, presumably because they can synthesize it (based on the pathway analysis, Figure 4C).

### Influences of parasitism on host amino acid synthesis, gene expression, and free amino acid content in host hemolymph

Our comparative genomics analyses and feeding assays have showed that *C. chilonis* has lost the ability to synthesize eight amino acids that are essential for parasitoid survival. The next step was to test whether these eight amino acids were available in host hemolymph, and if concentrations were altered in parasitized host hemolymph. To this end, we conducted a metabolomic analysis of the fourth-instar larval hemolymph of *C. suppressalis*. In the non-parasitized *C. suppressalis* larvae, all eight amino acids were represented in the hemolymph. Histidine was the most abundant at a concentration of 4.455 mg/ml, followed by glutamine at a concentration of 3.262 mg/ml (Figure 5A). In the parasitized larvae, the amounts of four amino acids (arginine, serine, tyrosine, and alanine) were significantly increased and four amino acids (5-hydroxylysine, glutamic acid, methionine, and lysine) were significantly decreased in the first 3 days after parasitism (p<0.05, Student's *t*-test). Among the eight amino acids that *C. chilonis* cannot synthesize by itself, lysine was found to be significantly decreased in the host hemolymph in the first 3 days after parasitism, likely resulting from the absorption of lysine by the wasp larvae. However, tyrosine was significantly increased in the first 3 days after parasitism, while levels of six other amino acids (valine, tryptophan, histidine, phenylalanine, isoleucine, and leucine) were not significantly changed in the hemolymph. These findings suggest that parasitism by *C. chilonis* manipulates the *C. suppressalis* larvae to store or release amino acids into the hemolymph, possibly for the first instar larvae of *C. chilonis* to absorb the free amino acids, such as lysine, from the host hemolymph (Figure 5A).

**Figure 5.** Parasitism by *C. chilonis* influences the host amino acid synthetic pathway and free amino acid levels in host hemolymph. (**A**) Free amino acids levels in host hemolymph were changed after parasitism. UPLC-MS/MS analysis was used. Host hemolymph was collected 3 days after parasitism. The detection for each treatment were repeated 10 times. Student’s *t*-test was used for statistical analysis of amino acid changes. (**B**) Gene expression of amino acid biosynthetic pathways was changed 2 days after parasitism. Black line indicates the reaction exists in host, while grey line indicates the interaction cannot be found. Up- and down-regulated genes were considered if there was a fold change ≥2 and p-adjusted <0.05 in host fat body and hemocyte transcriptome data. Only the genes with significantly expression changes are showed. The asterisk indicates that the concentration of amino acids was significantly changed three days after parasitism. *Significant difference at p<0.05, **at p<0.01. Figure 5—source data 1.This table includes the free amino acids levels in host hemolymph. Figure 5—source data 2.This table includes the host’s differentially expressed genes of amino acid biosynthetic pathways after parasitism.

**Figure 5—figure supplement 1.** Influence of parasitism on gene expression of the amino acid biosynthetic pathways in fat body and hemocytes of the host *C. suppressalis*.

Next, we used the previously reported transcriptome of host fat body and hemolymph in unparasitized and post-parasitized hosts to examine differential gene expression (Wu et al., 2013). It was found that 16 protease genes were significantly upregulated (4–59-fold) in fat body and hemolymph of the host following parasitism (Supplementary file 2 – Table 6). Most were the genes encoding serine proteases, trypsins and carboxypeptidases, which play important roles in proteolysis. These data suggest that parasitoid wasps can stimulate the expression of key proteases in the host to help hydrolyze proteins to free amino acids. In addition, parasitism does not have significant influence on host’s amino acid biosynthetic pathways, as the expression of most genes (82%) in the pathways were not changed significantly after parasitism (Figure 5B, Figure 5—figure supplement 1). Only six genes were found to be significantly downregulated in the fat body. Interestingly, we found that five genes in the amino acid biosynthetic pathway were significantly upregulated after parasitism. All of them are also belong to glycolysis (M00002) and citrate cycle (M00010) (Figure 3B). This finding indicates that parasitism may activate the host’s carbohydrate metabolism. Our results suggest that *C. chilonis* venom and/or larvae feeding may finely regulate the host’s protease activity to re-allocate the amino acids into the hemolymph, to ensure adequate nutrition for the parasitoid. However, we have so far not been able to separate the effects of venom from actions of feeding larvae in this endoparasitoid wasp.

### Amino acid transport in the parasitoid wasp *C. chilonis*

We also explored the repertoire of amino acid transporters, which recognize and transport free amino acids across the plasma membranes of animal cells (Wolfersberger, 2000). The free amino acids in host hemolymph are absorbed by early instar larvae through both the gut epithelium and thin exoskeleton, and only through the gut epithelium in late-instar larvae (Giordana et al., 2003; Caccia et al., 2005; Grimaldi et al., 2006; Pennacchio et al., 2014). However, it is uncertain whether the amino acid absorption is correlated with enhanced transport ability. To investigate this possibility, we examined transporter gene families associated with amino acid transport, including ATP-binding cassette transporters (ABC transporters) and amino acid transporters (AATs). ABC transporters comprise an extensive and variable transporter superfamily and play a role in transferring a variety of compounds across cellular membranes, including amino acids, sugars, lipids, and other xenobiotics (Dermauw and Van Leeuwen, 2014). AATs are more specifically for transferring amino acids (Wolfersberger, 2000). In total, 103 ABC transporter genes were identified in the *C. chilonis* genome. Compared with other hymenopteran insects, the ABC transporters gene family showed expansion in *C. chilonis*, as revealed by maximum likelihood phylogenetic analysis (Figure 6A, Supplementary file 2 – Table 7). In contrast, M. demolitor, the closest relative of *C. chilonis* in our study, only has 51 ABC transporters in the genome. This result indicates that the expansion of ABC transporters occurred after divergence of *C. chilonis* and *M. demolitor* (Supplementary file 2 – Table 7). We found 36 ABC transporters were more highly expressed in the larval stage relative to the pupal stage (FoldChange (FPKM) >2). The amino acid/polyamine/organocation (APC) family and the amino acid/auxin permease (AAAP) gene family are closely associated with nutrition transport in insects (Colombani et al., 2003; Price et al., 2014). Ten putative APCs and eight putative AAAPs were identified in the C. chilonis genome (Supplementary file 2 – Table 8). Although phylogenetic analysis showed that the APC gene family was not significantly expanded, transcriptome analysis results indicate that two APC genes were highly expressed in the larval stage relative to the pupal and adult stages. Five APC genes were highly expressed in the larval and pupal stages relative to the adult stage (Figure 6B). However, only one AAAP gene was highly expressed in larvae (Figure 6—figure supplement 1). We next searched for these transporter genes in a large collection of hymenopteran genomes, but the results did not support the view that these transporter genes are expanded basally in the parasitoid wasps (Figure 6—figure supplement 2). This finding suggests that the expansion of ABC transporters in *C. chilonis* is an independent event, as it was not found in close relatives. The expansion events also independently occurred in the sawfly *Cephus cinctus*, some ants, *Megachile* bees and *Bombus* bees. Interestingly, some host amino acid transporters, such as vacuolar amino acid transporters, vesicular glutamate transporters, and proton-coupled amino acid transporter-like proteins, were significantly upregulated after parasitism (Supplementary file 2 – Table 9). These data show that the amino acid transport ability in *C. chilonis* may be significantly enhanced by gene family expansion and increased expression. Upregulation of host genes involved in amino acid transport could contribute to release free amino acids into the hemolymph, and therefore their role in amino acid availability for parasitoid larvae warrants future investigation.

**Figure 6.** Amino acid transport genes in parasitoid wasp *C. chilonis*. (**A**) ABC transporter genes of *C. chilonis*. A total of 103 ABC transporter genes were identified in the *C. chilonis* genome. The ABC transporter gene family was significantly expanded in *C. chilonis* as revealed by phylogenetic comparison with the honeybee *A. mellifera* and the sawfly *A. rosae*. Heatmap showed the expression patterns of these 103 ABC transporter genes at different developmental stages. (**B**) Amino acid/polyamine/organocation (APC) family of *C.* c*hilonis*. A total of 10 APC genes were found in *C. chilonis* genome. Phylogenetic analysis showed APCs were not expanded in *C. chilonis* compared with honeybee and sawfly. Transcriptome analysis showed 7 APCs were highly expressed at both larval and pupal stages, suggesting the amino acid transport ability was active at these two development stages. Yellow represents higher expression values while dark blue represents lower expression. Figure 6—source data 1.This file includes the phylogeny tree file of ABC transporter genes in Figure 6A. Figure 6—source data 2.This file includes the phylogeny tree file of APC genes in Figure 6B. Figure 6—source data 3.This file includes the gene expression levels (FPKM) of ABC transporter genes in *C. chilonis*. Figure 6—source data 4.This file includes the gene expression levels (FPKM) of APC genes in *C. chilonis*.

**Figure 6—figure supplement 1.** Phylogenetic relationships of the AAAP family and gene expression in *C. chilonis* at different development stages.

**Figure 6—figure supplement 2.** Number of predicted ABC transporter genes, APC family and AAAP family across hymenopteran lineages.

## Discussion

Our original motivation for this study was to investigate amino acid pathway gene loss in the parasitoid Hymenoptera, with the expectation that they would show greater loss rates than other hymenopterans, due to their amino-acid-rich diet. This expectation was not met. Rather we detected major pathway losses basally in the Hymenoptera (and Holometabolous insects), and additional amino acid losses scattered independently in both the aculeates and parasitoids, without strong evidence of an accelerated rate in Parasitoida. More extensive whole genome sequencing will help reveal what ecological and dietary features may be associated with these losses, as well as potential roles for associated microbiomes as sources for amino acids.

Our comparative pathway analysis shows that hymenopterans’ loss of biosynthetic capability for several amino acids was caused by degradation of one or several key genes in the relevant pathways, and this trait loss occurs in both parasitoid wasps and aculeate species (Figure 2, Supplementary file 1 – Table 1). However, the majority of amino acid synthesis losses occurred basally in the holometabolous insects and early in hymenopteran evolution. Trait loss is widely reported across diverse taxonomic groups, and can occur when their ecologically associated species (e.g. prey, plants, or microbial symbionts) provide the necessary resources or functions (Ellers et al., 2012).

Gene losses have been identified in amino acid biosynthesis pathways for other insects, such as ants, aphids, planthoppers, and mealybugs, indicating that gene loss in amino acid biosynthesis pathways is relatively common for insects. However, these gene losses may be due to very different factors in different organisms. For example, almost all phloem-sapping insects cannot synthesize some essential amino acids, but rely on endosymbionts for nutrition compensation (Douglas, 2006; McCutcheon and Moran, 2007; Douglas, 2009; Richards et al., 2010; Feldhaar, 2011; Xue et al., 2014; Husnik and McCutcheon, 2016; Gil et al., 2018). In contrast to phloem-sapping insects, which feed on a nutrient-poor diet, parasitoid wasps receive a diet rich in proteins and lipids from their host. Previous studies showed the lack of lipogenesis in most parasitoid wasps (Visser and Ellers, 2008; Visser et al., 2010). However, no extensive losses of genes involved in lipogenesis were noted (Visser et al., 2012; Lammers et al., 2019). In this study, we found that all hymenopterans appear to lack the capability to synthesize seven amino acids (four were lost earlier in holometabolous insects and three were lost in the common ancestor of Hymenoptera), and some parasitoids and aculeates have additionally lost the capability to synthesize lysine. The trait loss of lysine biosynthesis in parasitoid wasps may implicate their amino-acid-rich diet combined with the capability of parasitoids to manipulate the nutritional quality of hosts through venoms and other means. The trait loss in aculeates also may reflect their specialized diets. For example, bees feed on amino acid rich pollen and ants have a wide range of food sources (Rabie et al., 1983; Nicolson and Human, 2013). Another possibility is that symbiotic bacteria can provide essential nutrients to host insects, as reported in *Cephalotes* ants by Hu et al., 2018 and as well known in other insects such as aphids (Wilson et al., 2010; Feng et al., 2019).

Previous studies indicate that intracellular bacteria *Buchnera* (symbiotic bacteria of aphids) significantly contributes to parasitoid host nutritional suitability (Pennacchio et al., 1999; Rahbé et al., 2002). In our study, the synthesis capability of lysine was found to be lost in the common ancestor of two aphid parasitoids *A. ervi* and *L. fabarum*. This phenomenon may be associated with their parasitoid relationship with aphids, which possess intracellular bacteria that provide amino acids to the host (Wilson et al., 2010; Feng et al., 2019). Further study is needed to extend taxon sampling and determine how amino acid synthetic pathways have evolved in aphid parasitoids, as well as how they have evolved in other parasitoid-host-symbiont systems (e.g. parasitoids of mealybugs). Also, it would be interesting to study how they have evolved in plant-feeding members of the Parasitoida (e.g. fig wasps) (Xiao et al., 2013; Peters et al., 2017). We also point out that our conclusions are based on the canonical amino acid synthesis pathways that have been characterized (Kanehisa et al., 2017). We cannot rule out that unidentified pathways exist in insects that can ‘rescue’ individual amino acid biosynthesis, or that some genes have evolved so quickly that they are no longer recognized as canonical amino acid synthesis genes.

Parasites are ubiquitous in nature, and nutrition exploitation is one of the most important aspects of parasitism (Pennacchio et al., 2014). Understanding the genetic basis of nutrition exploitation by parasitoid insects can be of importance for understanding the parasitism strategy and also for customizing an artificial diet to rear parasitoids for use in biological control. Previous studies have reported that parasitism can alter the host’s metabolic system and release nutrients into hemolymph to increase nutritional suitability for parasitoid through venoms, teratocytes and parasitoid larval feeding (Digilio et al., 2000; Nakamatsu and Tanaka, 2003; Nakamatsu and Tanaka, 2004; Caccia et al., 2005; Falabella et al., 2005; Falabella et al., 2007; Falabella et al., 2009; Caccia et al., 2012; Mrinalini et al., 2015). Many previous studies have demonstrated in vitro that some essential amino acids, which are of considerable importance in the nutritional and metabolic adaptations of parasitoid wasps, are supplied by the host (Giordana et al., 2003; Caccia et al., 2005). Here, we present genome-level evidence that *C. chilonis* has lost the capability for de novo biosynthesis of eight amino acids. Among these eight amino acids, the capability to synthesize four amino acids (histidine, tryptophan, tyrosine, and phenylalanine) was lost early in holometabolous insects, prior to divergence of the basal Hymenoptera. The synthetic capability of additional three amino acids (valine, leucine and isoleucine) was subsequently lost in the common ancestor of Hymenoptera. The capability to synthesize lysine was lost in the common ancestor of *Cotesia*, *Microplitis* and *Macrocentrus* (Figure 2). This was also confirmed in vitro by rearing *C. chilonis* larvae in the medium deleting one or more specific amino acids. In addition, we noted significant increases in the number of amino acid transporter genes in *C. chilonis* (Figure 6), although the biological significance of this finding remains unclear. Our results are consistent with previous studies on the requirements of essential amino acids for parasitoid wasps and also explained why parasitoid wasps cannot survive on the chemically defined media without one or more kinds of these critical nutrients (Thompson, 1976; Thompson, 1981; Thompson, 1986; Bale et al., 2008). The metabolomic analysis showed that parasitism by *C. chilonis* significantly changed the levels of various amino acids in host hemolymph (Figure 5A). For the eight amino acids that *C. chilonis* cannot synthesize, the concentrations of lysine and tyrosine were found to change significantly in host hemolymph after parasitism (tyrosine went up, lysine went down). This result suggests that early larvae parasitoids may largely absorb lysine in host hemolymph, since lysine is essential for parasitoid development. In addition, venom and/or other effectors produced by parasitoids (i.e. PDV, teratocytes), and/or by larvae feeding significantly increase the concentration of tyrosine in host hemolymph, but parasitoid larvae utilize only a small amount of tyrosine at early stages (3 days after parasitism). These interpretations are speculative, and would require further detailed analysis to determine the contributions of modifications induced by wasp venom, teratocytes, and feeding larvae on amino acid levels.

Based on results from previous studies of the same parasitoid-host system (Hang and ZQ, 1991), it is likely that parasitism first increases amino acid levels in host hemolymph, then newly hatched wasp larvae begin to absorb and consume these amino acids and continue to do so at specific times during their development. To build a bigger picture of how parasitoid influence the amino acid levels in host hemolymph, more intensive sampling is required. The roles of venoms, PDV, teratocytes, and larval feeding in nutrition exploitation of *C. chilonis* in amino acid production need to be explored in the future.

Many parasitoid wasps are important natural enemies of agriculture and forestry pests and have been used as biological control agents for a long time (Quicke, 1997; Beckage and Gelman, 2004), such as Trichogrammatid wasps (Knutson, 1998; Lindsey et al., 2018). The use of artificial diets for mass rearing of parasitoids is an important aspect of increasing their utility and cost effectiveness for augmentative biological control. With the results in this study, we provide information on which amino acids need to be supplemented to artificial diets according to the pathway completeness of each parasitoid wasp. The approach suggests one utility of parasitoid genome sequences in advancing cost-effective biological control methods.

In summary, comparative genomic analysis of two superfamilies of parasitoid wasps, non-parasitoid hymenopterans (sawflies, paper wasps, ants, and bees), seven additional holometabolous insects in three orders, and six more basal arthropods provides genome-wide evidence that the synthesis capability for tryptophan, phenylalanine, tyrosine, and histidine was lost in holometabolus insects prior to hymenopteran divergence, and the synthesis capability of valine, leucine, and isoleucine predicted by pathway analysis was lost in the common ancestor of Hymenoptera. Loss of synthesis capability of lysine subsequently occurs during the Hymenoptera evolution by independent pathway disruptions. The loss of synthesis capability of amino acids was demonstrated by amino acid depletion feeding assays in *C. chilonis*. Metabolomic analysis provides an explanation that the required nutritional resource of parasitoid wasps is increased in parasitized host insects through host manipulation by venoms, teratocyte and/or parasitoid larval feeding. Expansion of amino acid transporters and their increased expression in the larval stage indicate that they might play important roles in nutrition interaction between parasitoid and host; however, this has not been as extensively investigated. Our finding also provides key information for designing artificial diets for mass-production of parasitoids as cost-effective biological control agents.

## Materials and methods

### Insect rearing

The parasitoid wasp *C. chilonis* and its host *C. suppressalis* were initially collected from fields in the experimental farmland of Zhejiang University, Hangzhou, China in 2012, and reared under laboratory conditions as previously described (Teng et al., 2016; Teng et al., 2017). Both laboratory colonies were maintained in an environmental chamber with constant conditions of 28 ± 1°C, about 70% RH and 16 L: 8 D photoperiod.

### Genome sequencing and assembly

Adopting a whole-genome shotgun sequence strategy and next-generation sequencing technologies, we used Illumina HiSeq 2000 and Pacbio platforms to sequence the genome of *C. chilonis*, supported by Novogene Bioinformatics Institute (Beijing, China). DNA was extracted from 300 haploid third-instar male wasp larvae. We prepared sequencing libraries with insert sizes of 250 bp, 2 Kb, 5 Kb, and 10 Kb for paired-end reads. Finally, we generated about 64.44 Gb of Illumina reads and 7.63 Gb of Pacbio reads (~380 X coverage, Supplementary file 2 – Table 10). Based on Overlap-Layout-Consensus, we de novo assembled the genome with Pacbio data. Then, we used PILON software (Walker et al., 2014) for error correction with Illumina data. Finally, the consensus sequences were assembled to the genome using SSPACE software (version 3) (Boetzer et al., 2011). The final assembly yielded 189 Mb of the reference genomic sequence with a scaffold N50 of 2.2 Mb.

### Transcriptome sequencing

In total, we sequenced six transcriptomes for assisting genome annotation and further analysis. Total RNA was isolated from early larvae (3 days after parasitism), later larvae (9 days after parasitism), male pupae, female pupae, male adults, and female adults of *C. chilonis* using the TRIzol protocol (Life Technologies, USA). RNA sequencing libraries were constructed using the Illumina mRNA-Seq Prep Kit (Illumina, USA). Briefly, oligo (dT) magnetic beads were used to purify poly(A)-containing mRNA molecules. The mRNA was further fragmented and randomly primed during first-strand synthesis by reverse transcription. This procedure was followed by second-strand synthesis with DNA polymerase I to create double-stranded cDNA fragments. The double-stranded cDNA was subjected to end repair by Klenow and T4 DNA polymerases, and A-tailed by Klenow lacking exonuclease activity. We then ligated the cDNA to Illumina Paired-end Sequencing adapters, performed size selection by gel electrophoresis, and then PCR amplification to complete library preparation. The libraries were sequenced using Illumina HiSeq 2000 (101 bp at each end). The RNA-seq reads were either de novo assembled using Trinity (Haas et al., 2013) or mapped to the *C. chilonis* genome using HISAT2 (Kim et al., 2015) with default parameters.

### Genome assembly assessment

We ran the core eukaryotic genes mapping approach (CEGMA) (version 2.4) to estimate the gene space (Parra et al., 2007), showing that 237 (95.6%) out of 248 CEGMA genes were represented in the genome assembly. Evaluation using Benchmarking Universal Single-Copy Orthologs (BUSCO) (version 3)confirmed the high quality of genome assembly (Simão et al., 2015), showing that 96.6% of 1658 Single-Copy BUSCOs (insecta_odb9) were complete in length (Supplementary file 2 – Table 11). Default parameters of CEGMA and BUSCO software were used.

### Genome annotation

The *C. chilonis* genome was annotated using the OMIGA genome annotation pipeline (OMIGA) (Liu et al., 2014), which is an optimized Maker-based insect genome annotation workflow. First, we identified repeat sequences. The repeat library was constructed using RepeatModeler software (version 1.0.7). Transposable elements (TEs) were predicted in the assemblies by homology searching against RepBase using RepeatMasker software (version 4.0.5) (Tempel, 2012) with default parameters. In total, we predicted 353,649 repeat sequences in a total of 68 Mb, which constitutes 36.18% of the *C. chilonis* genome (Supplementary file 2 – Tables 11–12). Second, we mapped RNA-seq raw data to the genome. Six transcriptomes from different development stages were applied as the evidence of gene expression. Trimmomatic software (version 0.36) (Bolger et al., 2014) was used for quality filtering of all the RNA-seq raw data, then Bowtie software (version 2.2.5) (Langmead et al., 2009) was used to map RNA-seq data to the genome. Next, we used HISAT2 (Kim et al., 2015) and StringTie (version 1.3.4) (Pertea et al., 2015) to obtain putative transcripts (Pertea et al., 2016). Default parameters were used for all the above programs.

To ensure high accuracy of gene prediction, we re-trained the de novo gene prediction software before genome annotation. We selected transcripts from the StringTie genes for training. TransDecoder (version 2.0.1) was used to identify candidate-coding regions in transcript sequences. To improve sensitivity, we also applied BLAST against UniProtKB/Swiss-Prot proteins (*E* < 10^−5^) and searched Pfam to identify protein domain information (*E* < 10^−5^). Only genes with complete ORFs were regarded as candidates. If a gene had multiple transcripts, only the longest was chosen. After TransDecoder software filtering, the gene candidates were used to re-train the Augustus (version 3.1) (Stanke et al., 2004) and SNAP (version 2006-07-28) (Korf, 2004) prediction software. For GeneMark-ET (Suite 4.21) (Lomsadze et al., 2014), more than 10 Mb of the genome sequence was used to re-train the software. The default parameters were used for training.

Three kinds of evidence were applied to annotate the protein-coding genes in the *C. chilonis* genome: homology-based predictions, de novo predictions and transcriptome-based predictions. MAKER pipeline (version 2.31) (Campbell et al., 2014) was used to annotate protein-coding genes of the *C. chilonis* genome. In the MAKER pipeline, sequences of homologous proteins from the NCBI invertebrate RefSeq were used. Three gene prediction programs including Augustus, SNAP and GeneMark-ET, which had all been re-trained, were used to predict coding genes. Additionally, the RNA-Seq data were mapped to the genome using HISAT2, and StringTie was used to assemble transcripts to the gene models. All gene sequences predicted from the above three approaches were combined by MAKER into a weighted and non-redundant consensus of gene structures. All the MAKER parameters were default settings. In total, OMIGA identified 14,142 protein-coding genes in the *C. chilonis* genome (Supplementary file 2 – Table 11).

### Ortholog analysis and comparative genomics

We used OrthoMCL (Li, 2003) to found orthologous groups from protein sequences of fourteen Hymenoptera insects (*A. rosae*, *O. abietinus*, *M. cingulum*, *M. demolitor*, *C. chilonis*, *D. alloeum*, *F. arisanus*, *C. floridanum*, *T. pertiosum*, *C. solmsi*, *N. vitripennis*, *S. invicta*, *A. cephalotes* and *A. mellifera*), of which the genome sequence data quality met the requirements for ortholog analysis, and one Coleoptera species (*T. castaneum*) (Supplementary file 2 – Table 13). We used the default parameters settings and identified 2291 single-copy protein-coding genes from 17,248 OrthoMCL clusters using a custom perl script. The distribution of pairwise amino acid identity was measured for each ortholog protein by the needle module in the EMBOSS packages (version 6.6.0) (Olson, 2002). In total, there were 6431 orthologs between *C. chilonis* and *A. mellifera*, 6596 orthologs between *C. chilonis* and *D. alloeum*, 6640 orthologs between *C. chilonis* and *F. arisanus*, 5902 orthologs between *C. chilonis* and *M. cingulum*, 7017 orthologs between *C. chilonis* and *M. demolitor*, 5908 orthologs between *C. chilonis* and *N. vitripennis*, 7114 orthologs between *C. floridanum* and *T. pretiosum*, 7104 orthologs between *N. vitripennis* and *C. solmsi*, 7554 orthologs between *A. cephalotes* and *S. invicta*, and 6810 orthologs between *A. mellifera* and *S. invicta*. These ortholog groups were used for pairwise amino acid identity analysis.

### Synteny analysis

We used the MCScanX software package (Wang et al., 2012) to perform synteny analysis between two pairs of braconid wasps including *C. chilonis* vs. *M. cingulum* and *C. chilonis* vs. *M. demolitor*. The scaffolds that contained more than five genes were considered for gene collinearity analysis. We found orthologous counterparts between the two pairs by BLASTP (*E* < 10^−10^). Specifically, syntenic blocks were defined when at least five orthologous counterparts were both clustered and located in continuous loci in a single scaffold for each species in each pair.

### Phylogenetic analysis

We reconstructed a phylogeny of 14 Hymenopteran and 1 Coleopteran species from genomic data, using 2291 single-copy protein-coding genes, and rooted on the red flour beetle *T. castaneum*.

The single-copy protein-coding genes were obtained from the OrthoMCL results. The protein sequences of single-copy protein-coding genes were aligned using MAFFT (version 7) (Katoh et al., 2002) with the default parameters. Then we filtered the saturated sites and poorly aligned regions using trimAl (Capella-Gutiérrez et al., 2009) and concatenated to one super-sequence for each species for the phylogenetic analysis.

The phylogenetic tree was reconstructed using RAxML (version 8.2.10) (Stamatakis, 2015), and IQ-TREE ModelFinder software (Kalyaanamoorthy et al., 2017) was used to select the best substitution model. Specifically, we used the ‘LG+I+F+G4’ model, and values of statistical support were obtained from 1000 replicates of bootstrap analysis. MCMCtree within the PAML software package (version 4.9 hr) (Yang, 1997) was used to estimate the divergence time between different species. Three calibration time points based on fossil records and previous studies, *Khutelchalcis gobiensis* (125.0–129.4 Mya), *Cretobraconus maculatus* (145.0–152.1 Mya), stem Hymenoptera (237.0–228.0 Mya), were used for divergence time calibration (Supplementary file 2 – Table 14).

### Gene family analysis

First, we obtained each gene family’s reference protein sequences from the GenBank of NCBI, and manually confirmed that each reference was intact and absolutely correct. Then, BLASTP was used to obtain the homolog candidate sequences with *E* < 10^−5^. All the candidate sequences were filtered by HMMER (Meng and Ji, 2013) (*E* < 10^−5^) against the Pfam database (Finn et al., 2016) to ensure each sequence contained the iconic domain structures characteristic of the gene family, and the remaining sequences were considered to be the corresponding genes. All multiple-sequence alignments were performed using the MAFFT, and conservation blocks trimmed using trimAl software. All phylogenetic relationship trees were constructed using RAxML software with the appropriate model, as selected by the ModelFinder software and bootstrap 1000.

### Amino acid metabolic network reconstruction and comparative analysis

For amino acid synthetic pathway evolution analysis in the Hymenoptera, we applied a pathway annotation pipeline to a large collection of hymenopteran genomes (38 genomes) and an expanded representation of outgroups (13 genomes) specifically to investigate patterns of the gene loss across major lineages of Hymenoptera (Supplementary file 1 – Table 1). First, to minimize the impact on this analysis of genome contamination with bacterial sequences in the assemblies, we used a modification of the pipeline to detect bacterial scaffolds and lateral gene transfers (originally developed by Wheeler et al., 2013 and subsequently refined as described in Furguson et al., 2020). Bacterial scaffold contamination containing amino acid synthesis genes was detected in *Cotesia vestalis* (GenBank accession number: LQNH00000000), *Diadromus collaris* (GenBank accession number: LQNJ00000000), *Ceratosolen solmsi* (GenBank accession number: ATAC00000000) and subsequently removed from the analysis. Then, a pathway annotation tool BlastKOALA v2.2 (Kanehisa et al., 2016) was used to identify genes in amino acid biosynthetic pathway (Pathway name: 01230 Biosynthesis of amino acids). Another pathway annotation tool iPathCons (Zhang et al., 2014) was used to confirm the results. To avoid missing genes during annotation, we used TBLASTN to scan genes in genome assembly with *E* < 10^−5^ and coverage above 75%. For *C. chilonis*, we also checked the PacBio long reads by TBLASTN using the same cut-off values. To avoid the miss-annotation of some rapidly evolve genes, we also used TBLASTN (*E* < 10^−5^) to check the genome assembly with a protein from closely related species as the reference sequence.

We reconstructed the hymenopteran phylogeny by joining three phylogenetic trees, two of them are from pervious researches (Branstetter et al., 2017; Peters et al., 2017) and one is from this study. Because of the absence of some of the taxa used in this study in the previously mentioned ones, we reconstructed a phylogenetic tree that contains all Parasitoida (Ichneumonid/Chalcidoid) species used here that have genome annotation information, sawfly *Athalia rosae*, wood wasp *Orussus abietinus*, paper wasp *Polistes dominula*, ants *Harpegnathos saltator* and *Ooceraea biroi*, and bee *Apis mellifera* based on 2923 single-copy proteins obtained from OrthoMCL using the MAFFT-trimAl-ModelFinder-RAxML pipeline (described in Phylogenetic analysis section of Materials and methods). The divergence time was estimated using MCMCtree based on five calibration time points with 95% confidence intervals from Peters et al., 2017, including the common ancestor of ant and bee (136–193 Mya), the common ancestor of ant, bee and vespid wasp (150–212 Mya), the common ancestor of chalcidoid wasps (105–159 Mya), the common ancestor of braconid wasps (116–177 Mya), and the common ancestor of Apocrita (203–276 Mya).

The pathway disruptions and gene losses were identified using a KEGG online tool, KEGG Mapper (https://www.kegg.jp/kegg/mapper.html), for all predicted pathway genes. We then documented independent pathway disruption and gene loss events in the Ichneumonid/Chalcidoid and Aculeata clades based on the genes involved and phylogenetic positions. To test whether pathway disruptions in amino acid biosynthesis were increased in the Ichneumonid/Chalcidoid clade compared to the Aculeate clade, we regraded the percent of branches in Parasitoida and Aculeata relative to the total of the two infraorders to generate a random expected proportion of disruption events if rates of disruption were the same in both infraorders, and then used Fisher’s exact test to perform the statistical test because of the small sample size (N = 14). The median value of the branch estimated by MCMCtree was used for branch length calculation. The online tool http://www.quantpsy.org/chisq/chisq.htm was used to calculate Chi-square values, using the custom expected frequencies for the gene loss calculations along branches. Amino acid biosynthetic capability was evaluated in terms of metabolic pathway completeness. The loss of synthesis capability to a particular amino acid occurs when all currently known synthetic pathways for the amino acid are disrupted.

We reconstructed the ancestral amino acid biosynthetic pathways for Hymenoptera and Holometabola by comparing with the pathway completeness of species in the outgroups. If a complete pathway was found in at least one of the holemetabolous insects, it was assumed to be present in the common ancestor of the Holometabola, and similarly for the common ancestor of the Hymenoptera. We then identified the pathways which have been disrupted in the common ancestor of Hymenoptera and Holometabola, respectively. To test if gene loss is more likely to occur in the disrupted pathway, we calculated a random expected proportion based on the gene number of each pathway in the ancestral state of Hymenoptera, then used Chi-square to perform the statistical test using custom expected frequencies for the gene loss event.

### Rearing *C. chilonis* larvae in vitro

Based on the protocols for rearing other parasitoid wasps (Thompson, 1976; Thompson, 1981), the chemically defined rearing media were prepared in our laboratory following the composition of Grace's Insect Medium (Thermo Fisher, catalog number: 11605; see detail components and concentrations at Supplementary file 2 – Table 15). All chemicals were obtained from Sigma Chemical Company (Shanghai, China). To verify the requirements for eight different amino acids of *C. chilonis*, we in vitro reared wasp larvae in the different mediums. The Grace's Insect Medium was used as a positive control, and the baseline medium which deleted eight amino acids (lysine, tryptophan, phenylalanine, tyrosine, leucine, isoleucine, valine, and histidine) that *C. chilonis* cannot synthesize was used as a negative control. Nine other mediums were formulated by deleting only one amino acid (including eight amino acids which *C. chilonis* cannot synthesize and one amino acid (glycine) which *C. chilonis* can synthesize). The deletion was accompanied by proportional increases in the quantity of all the remaining amino acids to maintain a constant amino acid level through adding a single amino acid, namely, glutamate, as described previously (Thompson, 1976; Thompson, 1981). Each artificial rearing medium was then sterilized by passing through a 0.22 mm filter (Merck Millipore Ltd.; Tullagreen, Carrigtwohill, Co. Cork, IRL). Each solution was then stored at −20°C until use.

The protocol for rearing parasitoid wasps in vitro was based on the methods used for *N. vitripennis* (Brucker and Bordenstein, 2012; Shropshire et al., 2016). For each tested rearing medium, the larvae of *C. chilonis* were collected by dissecting the parasitized *C. suppressalis* larvae, which were cleaned with 70% ethanol for surface sterilization 5 days after parasitism. Ten wasp larvae were transferred onto a 3 μm pore transwell polyester membrane (Costar; Corning Incorporated, Corning, NY, USA) after washing with 1 × phosphate buffer saline (PBS) three times. Then, the transwell insert was transferred to a well with 250 μl of rearing medium in a 24-well plate. All plates were stored in a sterile Tupperware box at 27 ± 1°C for the duration of the experiment. To confirm whether the larvae were alive, body movement, gut movement and body color were considered as criteria. The rearing experiments were replicated three times. Photos were also taken every day and the larvae body lengths were measured using ImageJ software (version 1.47).

### Metabolomics analysis for free amino acids in host hemolymph

Larvae of parasitized and non-parasitized *C. suppressalis* were surface-sterilized with 75% ethanol. Their prolegs were then cut with a pair of scissors and 30 µl of hemolymph was collected using micropipette tips and transferred into a 1.5 ml Eppendorf tube containing 10 μl saturated α-phenylthiourea (PTU). After a brief centrifugation, 20 µl supernatant of hemolymph without hemocytes was collected and mixed with 80 μl of pre-cooled methanol. The mixture was vortexed for 1 min. After overnight incubation at 4°C, the sample was centrifuged at 14,000 g for 15 min at 4°C. The resulting supernatant (10 µl) was diluted 20-fold with 50% aqueous acetonitrile and subsequently mixed with an equal volume of internal standard solution (ISs) (100 ng/ml in 50% aqueous acetonitrile) prior to UPLC-MS/MS analysis with 1 μl of injection volume.

The UPLC-MS/MS analysis was performed on a Waters Acquity UPLC system (Waters, Milford, MA) coupled to a Triple Quad 5500 tandem mass spectrometer (AB Sciex, Framingham, MA), and 3 μl of each sample or calibration curve sample was injected onto a Waters BEH Amide column (100 mm ×2.1 mm, 1.7 μm) at a flow rate of 0.4 ml/min. The mobile phase consisted of (A) water with 10 mM ammonium formate and 0.2% formic acid and (B) acetonitrile with 2 mM ammonium formate and 0.2% formic acid. The chromatographic separation was conducted with a gradient elution program as follows: 0 min, 90% B; 0.5 min, 90% B; 5.5 min, 75% B; 6.5 min, 50% B; 7.5 min, 50% B; 7.51 min, 90% B; 10 min, 90% B. The column temperature was maintained at 40°C.

The samples eluted from the column were ionized in an electrospray ionization source in positive mode (ESI+). Source temperature: 550°C, curtain gas (CUR): 35 psi, ion source gas 1 (GS1): 50 psi, ion source gas 2 (GS2): 50 psi, collision gas (CAD): 8 psi, ion spray voltage (IS): 5500 V, entrance potential (EP): 10 V, collision cell exits potential (CXP1): 10 V. The scheduled multiple reaction monitoring (sMRM) was used to acquire data in optimized MRM transition (precursor >product), declustering potential (DP), and collision energy (CE) as shown in Supplementary file 2 – Table 16. The test samples and standard curve samples were analyzed simultaneously. AB Sciex Analyst software (version 1.5.2) was used to control instruments and acquire data.

### Transcriptome analysis and differential expression analysis

We followed the standard protocol of differential gene and transcript expression analysis of RNA-seq experiments with HISAT2 and StringTie (Pertea et al., 2016). First, we used Trimmomatic to remove adapter and low-quality sequences in RNA-seq raw data. We then mapped the sequences to the genome using Bowtie. We used HISAT2 and StringTie to obtain putative transcripts. Raw counts for each predicted gene were derived from the read alignments and normalized to fragments per kilobase of exon model per million mapped fragments (FPKM) and differential expression analyses were performed using RSEM (version 1.3.0) (Li and Dewey, 2011). Heatmaps were generated using R and the package pheatmap v1.0.8. Differentially expressed genes were identified using edgeR (version 3.11) (Robinson et al., 2010). Benjamini-Hochberg correction was used to adjust p values for multiple testing (FDR adjusted). We defined the fold change of gene expression ≥2 and p-adjusted <0.05 as the criteria for significantly differential expression changes.

## Data Availability

All sequence data of the *C. chilonis* genome project have been deposited in GenBank under the accession code RJVT00000000. In addition, all the data in this paper have been deposited in the InsectBase (www.insect-genome.com/cotesia/). The following dataset was generated: YeXXiongSTengZFangQWerrenJHYeGLiF2020Genome of C. chilonisNCBI BioProjectPRJNA501840 The following previously published datasets were used: WuSFSunFQiYYaoYFangQHuangJStanleyGYeG2013Parasitization by Cotesia chilonis influences gene expression in fatbody and hemocytes of Chilo suppressalisNCBI SRASRR65104010.1371/journal.pone.0074309PMC378108824086331 HallABPapathanosP-ASharmaAChengCAkbariOSAssourLBergmanNHCagnettiACrisantiADottoriniTFiorentiniEGaliziRHnathJJiangXKorenSNolanTRaduneDSharakhovaM VSteeleA2015Radical remodeling of the Y chromosome in a recent species radiationNCBI GenBankLCWJ00000000.110.1073/pnas.1525164113PMC483940927035980 KelkarYD2018Flesh Fly genome submissionNCBI GenBankQOCX00000000.1 HoskinsRACarlsonJWWanKHParkSMendezIGalleSEBoothBWPfeifferBDGeorgeRASvirskasRKrzywinskiRScheinJAccardoMCDamiaEMessinaGMéndez-LagoMde PablosBDemakovaOVAndreyevaENBoldyrevaLVMarraMCarvalhoBADimitriPVillasanteAZhimulevIFRubinGMKarpenGHCelnikerSE2015The Release 6 Reference Sequence of the Drosophila melanogaster GenomeNCBI AssemblyGCF_000001215.410.1101/gr.185579.114PMC435288725589440 LinY2019Chilo suppressalis genomeNCBI GenBankRSAL00000000.1 MitaKXiaQ2008The genome of a lepidopteran model insect, the silkworm Bombyx moriNCBI GenBankBABH00000000.119522291 MuraliSRichardsSBandaranaikeDBellairMBlankenburgKChaoHDinhHDoddapaneniHDugan-RochaSElkadiriSGnanaolivuRHernandezBSkinnerEJavaidMLeeSLiMMingWMunidasaMMunizJNguyenLHughesDOsujiNPuL-LPuazoMQuCQuirozJRajRWeissenbergerGXinYZouXHanYWorleyKMuznyDGibbsR2017Anoplophora glabripennis RefSeq Genome sequencingNCBI GenBankAQHT00000000.2 SaddBMBarribeauSMBlochGde GraafDCDeardenPElsikCGGadauJGrimmelikhuijzenCJHasselmannMLozierJDRobertsonHMSmaggheGStolleEVan VaerenberghMWaterhouseRMBornberg-BauerEKlasbergSBennettAKCamaraFGuigoRHoffKMariottiMMunoz-TorresMMurphyTSantesmassesDAmdamGVBeckersMBeyeMBiewerMBitondiMMBlaxterMLBourkeAFBrownMJBuechelSDCameronRCappelleKCarolanJCChristiaensOCiborowskiKLClarkeDFColganTJCollinsDHCridgeAGDalmayTDreierSdu PlessisLDuncanEErlerSEvansJFalconTFloresKFreitasFCFuchikawaTGempeTHartfelderKHauserFHelbingSHumann FCIrvineFJermiinLSJohnsonCEJohnsonRMJonesAKKadowakiTKidnerJHKochVKohlerAKrausFBLattorffHMLeaskMLockettGAMallonEBAntonioDSMarxerMMeeusIMoritzRFNairANapflinKNissenINiuJNunesFMOakeshottJGOsborneAOtteMPinheiroDGRossieNRueppellOSantosCGSchmid-HempelRSchmittBDSchulteCSimoesZLSoaresMPSweversLWinnebeckECWolschinFYuNZdobnovEMAqrawiPKBlankenburgKPCoyleMFranciscoLHernandezAGHolderMHudsonMEJacksonLJayaseelanJJoshiVKovarCLeeSLMataRMathewTNewshamIFNgoROkwuonuGPhamCPuLLSaadaNSantibanezJSimmonsDThorntonRVenkatAWaldenKKWuYQDebyserGDevreeseBAsherCBlommaertJChipmanADChittkaLFouksBLiuJO'NeillMPSumnerSPuiuDQuJSalzbergSLSchererSEMuznyDMRichardsSRobinsonGEGibbsRASchmid-HempelPWorleyKC2011The genomes of two key bumblebee species with primitive eusocial organizationNCBI GenBankAEQM00000000.210.1186/s13059-015-0623-3PMC441437625908251 PanHKapheimK2015The genome of Melipona quadrifasciataNCBI GenBankLIRP00000000.1 WallbergABunikisIPetterssonOVMosbechMBChildersAKEvansJDMikheyevASRobertsonHMRobinsonGEWebsterMT2018A hybrid de novo genome assembly of the honeybee, Apis mellifera, with chromosome-length scaffoldsNCBI GenBankQIUM00000000.210.1186/s12864-019-5642-0PMC645473930961563 PanHKapheimK2015The genome of Eufriesea mexicanaNCBI GenBankLLKC00000000.1 PanHKapheimK2015The genome of Habropoda laboriosaNCBI GenBankLHQN00000000.1 RobinsonGERobertsonHMHudsonMEWaldenKFischmanBJPitts-SingerTJamesRSalzbergSLPuiuDMagocTKelleyDZiminAV2011Megachile rotundata, whole genome shotgun sequencing projectNCBI GenBankAFJA00000000.1 PanHKapheimK2015The genome of Dufourea novaeangliaeNCBI GenBankLGHO00000000.1 NygaardSZhangGSchiottMLiCWurmYHuHZhouJJiLQiuFRasmusseMPanHHauserFKroghAGrimmelikhuijzenCJWangJBoomsmaJJ2011The genome of the leaf-cutting ant Acromyrmex echinatior suggests key adaptations to advanced social life and fungus farmingNCBI GenBankAEVX00000000.110.1101/gr.121392.111PMC314950021719571 SuenGTeilingCLiLHoltCAbouheifEBornberg-BauerEBouffardPCalderaEJCashECavanaughADenasOElhaikEFaveMJGadauJGibsonJDGraurDGrubbsKJHagenDEHarkinsTTHelmkampfMHuHJohnsonBRKimJMarshSEMoellerJAMunoz-TorresMCMurphyMCNaughtonMCNigamSOversonRRajakumarRReeseJTScottJJSmithCRTaoSTsutsuiNDViljakainenLWisslerLYandellMDZimmerFTaylorJSlaterSCCliftonSWWarrenWCElsikCGSmithCDWeinstockGMGerardoNMCurrieCR2011The genome sequence of the leaf-cutter ant Atta cephalotes reveals insights into its obligate symbiotic lifestyleNCBI GenBankADTU00000000.110.1371/journal.pgen.1002007PMC303782021347285 WurmYWangJRiba-GrognuzOCoronaMNygaardSHuntBGIngramKKFalquetLNipitwattanaphonMGotzekDDijkstraMBOettlerJComtesseFShihCJWuWJYangCCThomasJBeaudoingEPradervandSFlegelVCookEDFabbrettiRStockingerHLongLFarmerieWGOakeyJBoomsmaJJPamiloPYiSVHeinzeJGoodismanMAFarinelliLHarshmanKHuloNCeruttiLXenariosIShoemakerDKellerL2018The genome of the fire ant Solenopsis invictaNCBI GenBankAEAQ00000000.210.1073/pnas.1009690108PMC307841821282665 SmithCRSmithCDRobertsonHMHelmkampfMZiminAYandellMHoltCHuHAbouheifEBentonRCashECrosetVCurrieCRElhaikEElsikCGFaveMJFernandesVGibsonJDGraurDGronenbergWGrubbsKJHagenDEViniegraASJohnsonBRJohnsonRMKhilaAKimJWMathisKAMunoz-TorresMCMurphyMCMustardJANakamuraRNiehuisONigamSOversonRPPlacekJERajakumarRReeseJTSuenGTaoSTorresCWTsutsuiNDViljakainenLWolschinFGadauJ2010Draft genome of the red harvester ant Pogonomyrmex barbatusNCBI GenBankADIH00000000.110.1073/pnas.1007901108PMC307841221282651 RichardsSGibbsRAWeinstockGMBrownSJDenellRBeemanRWGibbsRBucherGFriedrichMGrimmelikhuijzenCJKlinglerMLorenzenMRichardsSRothSSchroderRTautzDZdobnovEMMuznyDAttawayTBellSBuhayCJChandraboseMNChavezDClerk-BlankenburgKPCreeADaoMDavisCChackoJDinhHDugan-RochaSFowlerGGarnerTTGarnesJGnirkeAHawesAHernandezJHinesSHolderMHumeJJhangianiSNJoshiVKhanZMJacksonLKovarCKowisALeeSLewisLRMargolisJMorganMNazarethLVNguyenNOkwuonuGParkerDRuizSJSantibanezJSavardJSchererSESchneiderBSodergrenEVattahilSVillasanaDWhiteCSWrightRParkYLordJOppertBBrownSWangLWeinstockGLiuYWorleyKElsikCGReeseJTElhaikELandanGGraurDArensburgerPAtkinsonPBeidlerJDemuthJPDruryDWDuYZFujiwaraHMaselliVOsanaiMRobertsonHMTuZWangJJWangSSongHZhangLWernerDStankeMMorgensternBSolovyevVKosarevPBrownGChenHCErmolaevaOHlavinaWKapustinYKiryutinBKittsPMaglottDPruittKSapojnikovVSouvorovAMackeyAJWaterhouseRMWyderSKriventsevaEVKadowakiTBorkPArandaMBaoRBeermannABernsNBolognesiRBonnetonFBoppDButtsTChaumotADenellREFerrierDEGordonCMJindraMLanQLattorffHMLaudetVvon LevetsowCLiuZLutzRLynchJAda FonsecaRNPosnienNReuterRSchinkoJBSchmittCSchoppmeierMShippyTDSimonnetFMarques-SouzaHTomoyasuYTraunerJVan der ZeeMVervoortMWittkoppNWimmerEAYangXJonesAKSattelleDBEbertPRNelsonDScottJGMuthukrishnanSKramerKJArakaneYZhuQHogenkampDDixitRJiangHZouZMarshallJElpidinaEVinokurovKOppertCEvansJLuZZhaoPSumathipalaNAltincicekBVilcinskasAWilliamsMHultmarkDHetruCHauserFCazzamaliGWilliamsonMLiBTanakaYPredelRNeupertSSchachtnerJVerleyenPRaibleFWaldenKKAngeliSForetSSchuetzSMaleszkaRMillerSCGrossmannD2014The genome of the model beetle and pest Tribolium castaneumNCBI GenBankAAJJ00000000.2 SmithCDZiminAHoltCAbouheifEBentonRCashECrosetVCurrieCRElhaikEElsikCGFaveMJFernandesVGadauJGibsonJDGraurDGrubbsKJHagenDEHelmkampfMHolleyJAHuHViniegraASJohnsonBRJohnsonRMKhilaAKimJWLairdJMathisKAMoellerJAMunoz-TorresMCMurphyMCNakamuraRNigamSOversonRPPlacekJERajakumarRReeseJTRobertsonHMSmithCRSuarezAVSuenGSuhrELTaoSTorresCWvan WilgenburgEViljakainenLWaldenKKWildALYandellMYorkeJATsutsuiND2011Draft genome of the globally widespread and invasive Argentine ant (Linepithema humile)NCBI GenBankADOQ00000000.110.1073/pnas.1008617108PMC307835921282631 McKenzieSKKronauerDJC2018The genomic architecture and molecular evolution of ant odorant receptorsNCBI GenBankQOIP00000000.110.1101/gr.237123.118PMC621164930249741 ShieldsEJShengLWeinerAKGarciaBABonasioR2018High-Quality Genome Assemblies Reveal Long Non-coding RNAs Expressed in Ant BrainsNCBI GenBankQANH00000000.110.1016/j.celrep.2018.05.014PMC602340429874592 PatalanoSVlasovaAWyattCEwelsPCamaraFFerreiraPGAsherCLJurkowskiTPSegonds-PichonABachmanMGonzalez-NavarreteIMinocheAEKruegerFLowyEMarcet-HoubenMRodriguez-AlesJLNascimentoFSBalasubramanianSGabaldonTTarverJEAndrewsSHimmelbauerHHughesWOGuigoRReikWSumnerS2014Molecular signatures of plastic phenotypes in two eusocial insect species with simple societiesNCBI GenBankJPHQ00000000.110.1073/pnas.1515937112PMC465316626483466 StandageDSBrendelVPTothAL2015Genome, transcriptome, and methylome sequencing of a primitively eusocial wasp reveal a greatly reduced DNA methylation system in a social insectNCBI GenBankLMBU00000000.110.1111/mec.1357826859767 HuangDWWangJCookJXiaoJHYueZJiaLYYangXHNiuLHWangZZhangPSunBFHeSMLiZXiongTLXinWGuHFWangBWerrenJWheelerDNiuLMMaGCTangTBianSNWangNXYangCYWangNFuYGMurphyRLiWZYiS.VYangXYZhouQLuCXXuCYHeLJYuLLChenMZhengYWangSWZhaoSLiYHYuYYQianXJCaiYBianLLZhangSWangJYYinYXiaoHWangGHYuHWuWS2013The fig wasp genome reflects extreme specialisation to a benign hostNCBI GenBankATAC00000000.1 WerrenJHRichardsSDesjardinsCANiehuisOGadauJColbourneJKWerrenJHBeukeboomLWDesplanCElsikCGGrimmelikhuijzenCJKittsPLynchJAMurphyTOliveiraDCSmithCDvan de ZandeLWorleyKCZdobnovEMAertsMAlbertSAnayaVHAnzolaJMBarchukARBehuraSKBeraANBerenbaumMRBertossaRCBitondiMMBordensteinSRBorkPBornberg-BauerEBrunainMCazzamaliGChaboubLChackoJChavezDChildersCPChoiJHClarkMEClaudianosCClintonRACreeAGCristinoASDangPMDarbyACde GraafDCDevreeseBDinhHHEdwardsRElangoNElhaikEErmolaevaOEvansJDForetSFowlerGRGerlachDGibsonJDGilbertDGGraurDGrunderSHagenDEHanYHauserFHultmarkDHunter HC IV HurstGDJhangianSNJiangHJohnsonRMJonesAKJunierTKadowakiTKampingAKapustinYKechavarziBKimJKiryutinBKoevoetsTKovarCLKriventsevaEVKucharskiRLeeHLeeSLLeesKLewisLRLoehlinDWLogsdon JMJrLopezJALozadoRJMaglottDMaleszkaRMayampurathAMazurDJMcClureMAMooreADMorganMBMullerJMunoz-TorresMCMuznyDMNazarethLVNeupertSNguyenNBNunesFMOakeshottJGOkwuonuGOPannebakkerBAPejaverVRPengZPrattSCPredelRPuLLRansonHRaychoudhuryRRechtsteinerAReeseJTReidJGRiddleMRobertsonHMRomero-SeversonJRosenbergMSacktonTBSattelleDBSchlunsHSchmittTSchneiderMSchulerASchurkoAMShukerDMSimoesZLSinhaSSmithZSolovyevVSouvorovASpringaufAStafflingerEStageDEStankeMTanakaYTelschowATrentCVattathilSVerhulstECViljakainenLWannerKWWaterhouseRMWhitfieldJBWilkesTEWilliamsonMWillisJHWolschinFWyderSYamadaTYiSVZecherCNZhangLGibbsRA2012Functional and evolutionary insights from the genomes of three parasitoid Nasonia speciesNCBI GenBankAAZX00000000.110.1126/science.1178028PMC284998220075255 YeXYeG2020A chromosome level genome assembly of the parasitoid wasp Pteromalus puparumNCBI GenBankVCDM00000000.210.1111/1755-0998.1320632562592 MuraliSRichardsSBandaranaikeDBellairMBlankenburgKChaoHDinhHDoddapaneniHDugan-RochaSElkadiriSGnanaolivuRHernandezBSkinnerEJavaidMLeeSLiMMingWMunidasaMMunizJNguyenLHughesDOsujiNPuL.-LPuazoMQuCQuirozJRajRWeissenbergerGXinYZouXHanYWorleyKMuznyDGibbsR2017Copidosoma floridanum Genome sequencingNCBI GenBankJBOX00000000.2 MuraliSRichardsSBandaranaikeDBellairMBlankenburgKChaoHDinhHDoddapaneniHDugan-RochaSElkadiriSGnanaolivuRHernandezBSkinnerEJavaidMLeeSLiMMingWMunidasaMMunizJNguyenLHughesDOsujiNPuL.-LPuazoMQuCQuirozJRajRWeissenbergerGXinYZouXHanYWorleyKMuznyDGibbsR2017Genome sequencing of Trichogramma pretiosum and its endosymbiontNCBI GenBankJARR00000000.2 GaoFGuQJPanJWangZH.YinCLLiFSongQSStrandMRChenXXShiM2016Cotesia vestalis teratocytes express a diversity of genes and exhibit novel immune functions in parasitismNCBI GenBankLQNH00000000.110.1038/srep26967PMC489058827254821 BurkeGRWaldenKKWhitfieldJBRobertsonHMStrandMR2015Widespread genome reorganization of an obligate virus mutualistNCBI GenBankAZMT00000000.210.1371/journal.pgen.1004660PMC416938525232843 YinCHuJLiF2017Genome analysis enriches our understanding of wasp parasitic tacticsNCBI GenBankMVJL00000000.1 RobertsonHMWaldenKKTvedteES.HoodGRFederJL.ForbesAALogsdonJMMcelroyKE2019Genome of the parasitoid wasp Diachasma alloeum, an emerging model for ecological speciation and transitions to asexual reproductionNCBI GenBankLDKA00000000.210.1093/gbe/evz205PMC678184331553440 GeibS2014Fari WGS AssemblyNCBI GenBankJRKH00000000.1 BIPAA2017Aphidius ervi genome v3.0BIPAAaphidius_ervi BIPAA2017Lysiphlebus fabarum genome v1.0BIPAAlysiphlebus_fabarum YeXWangZ2016Genomic analysis reveals new insights into parasitoid-host interactionNCBI GenBankLQNJ00000000.1 BIPAA2018Venturia canescens genome v1.0BIPAAventuria_canescens MuraliSRichardsSBandaranaikeDBellairMBlankenburgKChaoHDinhHDoddapaneniHDugan-RochaSElkadiriSGnanaolivuRHernandezBSkinnerEJavaidMLeeSLiMMingWMunidasaMMunizJNguyenLHughesDOsujiNPuL.-LPuazoMQuCQuirozJRajRWeissenbergerGXinYZouXHanYWorleyKMuznyDGibbsR2017Orussus abietinus isolate:OABI.00-Male Genome sequencing and assemblyNCBI GenBankAZGP00000000.2 LinnenC2019Neodiprion pinetum draft genomeNCBI GenBankSSWZ00000000.1 RobertsonHMRobinsonDEWannerKWaldenKKO2012The Genome of the Wheatstem Sawfly, Cephus cinctusNCBI GenBankAMWH00000000.1 MuraliSRichardsSBandaranaikeDBellairMBlankenburgKChaoHDinhHDoddapaneniHDugan-RochaSElkadiriSGnanaolivuRHernandezBSkinnerEJavaidMLeeSLiMMingWMunidasaMMunizJNguyenLHughesDOsujiNPuL.-LPuazoMQuCQuirozJRajRWeissenbergerGXinYZouXHanYWorleyKMuznyDGibbsR2017Athalia rosae genome sequencing and assemblyNCBI GenBankAOFN00000000.2 MuraliSRichardsSBandaranaikeDBellairMBlankenburgKChaoHDinhHDoddapaneniHDugan-RochaSElkadiriSGnanaolivuRHernandezBSkinnerEJavaidMLeeSLiMMingWMunidasaMMunizJNguyenLHughesDOsujiNPuL.-LPuazoMQuCQuirozJRajRWeissenbergerGXinYZouXHanYWorleyKMuznyDGibbsR2018Whole genome assembly of Oncopeltus fasciatus using multiple sequencing technologiesNCBI GenBankJHQO00000000.2 MoranNALiYPark H. SmithTE2019Chromosome-level assembly of the pea aphid genome using Hi-CNCBI GenBankSDIB00000000.110.1093/molbev/msz138PMC675907831173104 MuraliSRichardsSBandaranaikeDBellairMBlankenburgKChaoHDinhHDoddapaneniHDugan-RochaSElkadiriSGnanaolivuRHernandezBSkinnerEJavaidMLeeSLiMMingWMunidasaMMunizJNguyenLHughesDOsujiNPuL.-LPuazoMQuCQuirozJRajRWeissenbergerGXinYZouXHanYWorleyKMuznyDGibbsR2019Frankliniella occidentalis isolate:FOCC.00 Genome sequencingNCBI GenBankJMDY00000000.3 FaddeevaADerksMFAnvarYSmitSVan StraalenNRoelofsD2015The genome of Folsomia candidaNCBI GenBankLNIX00000000.1 LeeJ-SLeeB-YChoiB-S2018The genome of the water flea Daphnia magnaNCBI GenBankQYSF00000000.1 GrbicMVan LeeuwenTClarkRRombautsSRouzePGrbicVOsborneEDermauwWCao Thi NgocPOrtegoFHernandez-CrespoPDiazIMartinezMNavajasMSucenaEMagalhaesSNagyLPaceRDjuranovicSSmaggheGIgaMChristiaensOVeenstraJ.AEwerJMancilla VillalobosRHutterJ.LHudsonS.DVelezMYiSZengJPires-DaSilvaARochFCazauxMNavarroMZhurovVAcevedoGMijanovicAFawcettJ.ABonnetEMartensCBaeleGWisslerLSanchez-RodriguezATirryLBlaisCDemeestereKHenzSGregoryRMathieuJVerdonLFarinelliLSchmutzJLindquistEFeyereisenRVan de PeerY2011Genome assembly and annotation of the Tetranychus urticae genomeNCBI GenBankCAEY00000000.1

## Additional files

Supplementary file 1. Supplementary Table 1. Genes in amino acid biosynthetic pathways (KEGG map01230), '+' means present, 'x' means lost.

Supplementary file 2. Supplementary Tables 1 – 16.

Transparent reporting form
